The article "Vitamin D Receptor Gene Polymorphisms and Prognosis of Breast Cancer among African-American and Hispanic Women" was published in 2013. Journal: PLoS One.

# Vitamin D Receptor Gene Polymorphisms and Prognosis of Breast Cancer among African-American and Hispanic Women

**DOI:** 10.1371/journal.pone.0057967

**Published:** 2013-03-12

**Authors:** Dhruva K. Mishra, Yanyuan Wu, Marianna Sarkissyan, Suren Sarkissyan, Zujian Chen, Xiying Shang, May Ong, David Heber, H. Phillip Koeffler, Jaydutt V. Vadgama

**Affiliations:** 1 Division of Cancer Research and Training, Center to Eliminate Cancer Health Disparities, Department of Internal Medicine, Charles R. Drew University of Medicine and Science, Los Angeles, California, United States of America; 2 David Geffen UCLA School of Medicine, Los Angeles, California, United States of America; 3 UCLA-Jonsson Comprehensive Cancer Center, Los Angeles, California, United States of America; 4 Division of Hematology and Oncology, Cedars-Sinai Medical Center, UCLA School of Medicine, Los Angeles, California, United States of America; 5 National Cancer Institute of Singapore, National University, Singapore, Singapore; Queensland University of Technology, Australia

## Abstract

**Background:**

Vitamin D plays a role in cancer development and acts through the vitamin D receptor (VDR). Although African-Americans have the lowest levels of serum vitamin D, there is a dearth of information on VDR gene polymorphisms and breast cancer among African-Americans and Hispanics. This study examines whether VDR gene polymorphisms are associated with breast cancer in these cohorts.

**Methods:**

Blood was collected from 232 breast cancer patients (Cases) and 349 non-cancer subjects (Controls). Genotyping for four polymorphic variants of VDR (*FokI, BsmI, TaqI* and *ApaI*) was performed using the PCR-RFLP method.

**Results:**

An increased association of the VDR-Fok1 *f* allele with breast cancer was observed in African-Americans (OR = 1.9, p = 0.07). Furthermore, the FbTA, FbtA and fbtA haplotypes were associated with breast cancer among African-Americans (p<0.05). Latinas were more likely to have the VDR-ApaI alleles (*Aa or aa*) (p = 0.008). The VDR-ApaI *aa* genotype was significantly associated with poorly-differentiated breast tumors (p = 0.04) in combined Cases. Kaplan-Meier survival analysis showed decreased 5-year disease-free-survival (DFS) in breast cancer patients who had the VDR-Fok1 *FF* genotype (p<0.05). The Cox regression with multivariate analysis revealed the independent predictor value of the VDR-FokI polymorphism for DFS. The other three variants of VDR (*BsmI*, *TaqI* and *ApaI*) were not associated with disease outcome.

**Conclusions:**

VDR haplotypes are associated with breast cancer in African-Americans, but not in Hispanic/Latinas. The VDR-FokI *FF* genotype is linked with poor prognosis in African-American women with breast cancer.

## Introduction

Several studies have demonstrated a decrease in Vitamin D receptor (VDR) expression in breast cancer cells compared to normal breast cells [1]. Decreased levels of VDR in breast cancer cells could be due to VDR gene polymorphisms [2], and/or DNA methylation [3]–[5]. Alterations in VDR expression and activity could lead to deregulation of Vitamin D uptake, metabolism, and serum levels of biologically active Vitamin D.

VDR gene has multiple gene polymorphisms [6], and four important single nucleotide polymorphisms (SNPs) in exon 2 and 3′UTR region. These are VDR-FokI (rs2228570), VDR-BsmI (rs1544410), VDR-TaqI (rs731236) and VDR-ApaI (rs7975232). Functional studies have identified that the VDR-FokI polymorphism leads to a shorter VDR protein by altering a translation initiation site [7], [8]. Large meta-analyses have demonstrated a significant association of the VDR FokI polymorphisms with breast cancer [9], [10], and other cancers across multiple ethnic cohorts [11], [12]. The functional role of VDR-BSMI, VDR-TaqI, and VDR-ApaI, which are all located near the 3′UTR region, are not as clear. However, studies do suggest that these polymorphisms may alter the polyadenylation of the VDR mRNA transcript, and thus affect mRNA stability [13]. Several studies show contradictory results on these polymorphisms and risk for breast cancer. Some studies found an association of breast cancer with BsmI, TaqI and ApaI [14]–[18] polymorphisms while others found no associations [19]–[21].

We have examined four VDR polymorphisms (FokI, TaqI, BsmI, ApaI) in African-American and Hispanic women from South Los Angeles and their association with breast cancer risk and survival.

## Materials and Methods

### Ethics Statement

This study, including the consent protocol, was approved by the Charles R. Drew University of Science and Medicine Institutional Review Board (Approval # 00-06-041-13). Written informed consent was obtained from all participants.

### Study Population

This is a retrospective cohort hospital-based study. Subjects were selected from our current breast study database in the Division of Cancer Research and Training, at Charles R. Drew University of Medicine and Science. We selected 232 women with breast cancer as Cases (115 African-Americans and 117 Hispanic/Latinas), and 349 normal, healthy women as Controls (73 African-Americans and 276 Latinas). Subjects were recruited between 1995 and 2007, and had documented personal history, clinical history, and tumor pathology data.

### VDR polymorphisms

Genomic DNA was extracted from buffy coat samples using the Qiagen DNA extraction kit. Vitamin D receptor genotyping for all four single-nucleotide polymorphic sites (SNPs) was done by the PCR-RFLP method (polymerase chain reaction- restriction fragment length polymorphism analysis). We used the following flanking primers [16], [21]. The BsmI polymorphism was detected using one primer originating in exon 7 (Forward: 5′-CAACCAAGACTACAAGTACCGCGTCAGTGA-3′) and a second in intron 8 (Reverse: 5′-AACCAGCGGAAGAGGTCAAGGG-3′), amplifying an 823 base pair (bp) fragment spanning the BsmI site. The ApaI and TaqI polymorphisms were detected using one primer in intron 8 (Forward: 5′- AGAGCATGGACAGGGAGCAAG- 3′) and the other in exon 9 (Reverse: 5′-GCAACTCCTCATGGCTGAGGTCTCA- 3′), yielding a 745 bp fragment spanning the ApaI and TaqI site. VDR-FokI polymorphic site was amplified using following primers Forward -5′GATGCCAGCTGGCCCTGGCACTG3′ and Reverse – 5′ATGGAAACACCTTGCTTCTTCTCCCTC 3′. PCR conditions were as follows: denaturation at 94°C for 5 min, followed by 40 cycles of PCR at 94°C (30 sec), 60°C–63.5°C (30 sec), and 72°C (30 sec). Annealing temperature for BsmI, ApaI/TaqI and FokI PCR are 63.5°C, 61°C and 59.5°C, respectively. Following PCR, aliquots of the amplified PCR products was digested with BsmI, ApaI, TaqI and FokI in accordance with the manufacturer's specifications (New England Biolabs, Beverly, MA, USA). The presence (lowercase) or absence (uppercase) of the enzyme recognition site was identified by ethidium bromide staining of fragments separated in a 2% agarose gel. Genotypes were assigned as BB, Bb, bb for the BsmI polymorphisms, AA, Aa, aa for the ApaI polymorphisms, TT, Tt and tt for the TaqI polymorphisms and FF, Ff and ff for the VDR-FokI polymorphisms. For the BsmI cleaved PCR products, the single resultant fragment was 823 bp, whereas the two resultant fragments were 648 bp and 175 bp. The PCR products digested with TaqI enzyme resulted in fragments of 496 bp and 249 bp in the presence of the polymorphic cutting site. PCR products digested with ApaI enzyme result in fragments of 531 bp and 214 bp in the presence of the polymorphic cutting site. The PCR products of VDR-FokI polymorphism (273 bp) digested with FokI enzyme result in 198 bp and 75 bp products in the presence of restriction site.

### Statistical Analysis

We used SPSS (ver 11.5) software to analyze our data. The Pearson Chi-square test was used to determine the statistically significant differences in frequency distribution of VDR genotypes between Cases and Controls. If the Table had cells with a frequency less than 5, Fisher's exact test was utilized. The 2-sided exact p-value<0.05 was considered statistically significant. The deviation of distribution of VDR genotypes from Hardy-Weinberg equilibrium (HWE) was estimated using the web tool HWE Testing calculator, available online [22]. Associations between each VDR polymorphism and breast cancer was estimated using the Logistic Regression test at 95% confidence interval, and controlled for age and BMI. For each polymorphic site, the wild type genotype (FF, BB, AA, TT) was considered as the reference based on published literature. We also performed analysis of linkage disequilibrium (LD) between polymorphic sites in a locus, to identify “clusters” of highly correlated sites based on LD statistics. We calculated the haplotype frequencies and LD in Cases and Controls using the Haplotype software package available online [23], [24].

## Results

Table 1 shows the characteristics of subjects in the study. The mean age of African-American Cases and Controls is 52.9 and 50.7 years, respectively, and for Hispanic/Latinas Cases and Controls is 49.2 and 45.6 years, respectively. The mean BMI is >30 kg/m∧2. Among Cases, the distribution of histopathological characteristics between African-American and Hispanic women with breast cancer was similar (Table 1), and approximately ∼59.9% Cases had Stage I/II disease and 26.7% had Stage III/V disease. The majority of our patients had infiltrating ductal carcinoma (62.2%), moderately to poorly differentiated (>70%).

**Table 1:** Characteristics of Breast Cancer Cases and Controls.

Subject Characteristics	African-American	Latina	*P*-Value*
	(N = 188)	(N = 393)	
**Mean Age±SD (Range)**			
Cases	53±9	49±11	0.006
Controls	51±10	46±10	0.001
*P*-Value**	0.13	0.003	
**Mean BMI±SD (Range)**			
Cases	34±9	32±7	0.01
Controls	35±8	31±6	<0.001
*P*-Value**	0.74	0.19	
**Cases Only (N = 232)**	**N (%)**	**N (%)**	
***ER/PR Status***			
ER/PR+	60 (52)	54 (46)	0.24
ER/PR-	42 (37)	43 (37)	
Unknown	13 (11)	20 (17)	
***HER2 Status***			
3+	16 (14)	22 (19)	0.64
2+	12 (10)	14 (12)	
1+	27 (24)	21 (18)	
Negative	40 (35)	35 (30)	
Unknown	20 (17)	25 (21)	
**Histology**			
Infiltrating Ductal Carcinoma	72 (63)	72 (62)	0.77
Infiltrating Lobular Carcinoma	20 (17)	15 (13)	
Infiltrating Adenocarcinoma	4 (4)	2 (2)	
Infiltrating Intraductal Carcinoma	0 (0)	1 (1)	
Ductal	0 (0)	1 (1)	
Lobular	2 (2)	2 (2)	
Unknown	17 (15)	24 (2)	
**Differentiation**			
Well	10 (9)	6 (5)	0.23
Moderately	33 (29)	30 (26)	
Poorly	55 (48)	55 (47)	
Unknown	17 (15)	26 (22)	
**Stage**			
0	7 (6)	8 (7)	0.05
I	23 (20)	8 (7)	
II	46 (40)	47 (40)	
III	22 (19)	29 (25)	
IV	4 (4)	7 (6)	
Unknown	13 (11)	18 (15)	

* P-value<0.05 is significant.

** P-value assesses significance within the column. (P<0.05 is significant).

The VDR gene polymorphisms were genotyped in 188 African-American and 393 Hispanics/Latina women. No deviation was observed from Hardy-Weinberg equilibrium (HWE) in the genotypic distribution of the VDR-FokI, VDR-BsmI and VDR-ApaI polymorphisms in the study subjects. However, the VDR-TaqI distribution was not within HWE. Further analysis identified that the deviation of VDR-TaqI was contributed from Cases (p allele = 0.75, q allele = 0.25, χ^2^ = 13.52), but not from Controls (p allele = 0.79, q allele = 0.21, χ^2^ = 2.34) – data not shown.

Logistic regression analysis was also performed (adjusted for age and BMI) and showed no significant association of breast cancer with any of the VDR polymorphisms when all of the Cases were pooled together (Table 2). However, when the analysis was performed based on ethnic stratification of the African-American and Hispanic/Latina subjects, the VDR-FokI *Ff* genotype (OR = 2.2, 95% CI = 0.95-5.1, p = 0.06) and the *f* allele (OR = 1.9, 95% CI = 0.9-3.7, p = 0.07) showed an increased association with breast cancer among African-American subjects (Table 2) compared with the Hispanic/Latina subjects. In the Hispanic/Latina population, we found no significant difference in the frequency distribution of the VDR genotypes between Cases and Controls, and no association with any of the genotypes with breast cancer based on logistic regression analysis (Table 2).

**Table 2:** Distribution of VDR-FokI, VDR-BsmI, VDR-TaqI and VDR-ApaI genotypes in African-American and Hispanic/Latina Cases and Controls.

	All Subjects†				African-American Subjects††				Hispanic/Latina Subjects††			
	Control N (%)	Case N (%)	OR at 95% CI	* *P*-value	Control N (%)	Case N (%)	OR at 95% CI	* *P*-value	Control N (%)	Case N (%)	OR at 95% CI	* *P*-value
	N = 73	N = 115			N = 73	N = 115			N = 276	N = 117		
**VDR-FokI**												
FF	148 (42)	95 (41)	1.0		38 (52)	53 (46)	1.0		110 (40)	42 (36)	1.0	
Ff	144 (41)	110 (47)	1.3 (0.8–2.1)	0.26	30 (41)	55 (48)	2.2 (0.95–5.1)	0.06	114 (41)	55 (47)	1.0 (0.5–1.8)	0.98
ff	57 (16)	27 (12)	1.3 (0.7–2.6)	0.43	5 (7)	7 (6)	2.9 (0.3–26.3)	0.33	52 (19)	20 (17)	1.0 (0.5–2.2)	0.91
F allele	440 (63)	300 (64)	1.0		106 (73)	161 (70)	1.0		334 (61)	139 (59)	1.0	
f allele	258 (37)	164 (35)	1.2 (0.9–1.7)	0.29	40 (27)	69 (30)	1.9 (0.9–3.7)	0.07	218 (40)	95 (41)	1.0 (0.7–1.5)	0.92
**VDR-BsmI**												
BB	26 (7)	19 (8)	1.0		8 (11)	9 (8)	1.0		18 (7)	10 (9)	1.0	
Bb	141 (40)	90 (39)	0.8 (0.3–1.9)	0.57	31 (43)	40 (35)	0.7 (0.1–3.6)	0.63	110 (40)	50 (43)	0.9 (0.3–2.4)	0.76
bb	182 (52)	123 (53)	0.9 (0.3–1.9)	0.59	34 (47)	66 (57)	1.4 (0.3–7.9)	0.68	148 (54)	57 (49)	0.6 (0.2–1.7)	0.34
B allele	193 (28)	128 (28)	1.0		47 (32)	58 (25)	1.0		146 (26)	70 (30)	1.0	
b allele	505 (72)	336 (72)	0.9 (0.7–1.3)	0.76	99 (68)	172 (75)	1.6 (0.9–2.9)	0.15	406 (74)	164 (70)	0.75 (0.5–1.1)	0.19
**VDR-TaqI**												
TT	223 (64)	141 (61)	1.0		40 (55)	66 (57)	1.0		183 (66)	75 (64)	1.0	
Tt	106 (30)	66 (28)	0.8 (0.5–1.3)	0.31	28 (38)	35 (30)	0.6 (0.3–1.4)	0.24	78 (28)	31 (27)	0.9 (0.5–1.6)	0.66
tt	20 (6)	25 (11)	1.3 (0.5–3.0)	0.58	5 (7)	14 (12)	1.1 (0.3–4.4)	0.91	15 (5)	11 (9)	1.4 (0.5–4.0)	0.59
T allele	552 (79)	348 (75)	1.0		108 (74)	167 (73)	1.0		444 (80)	181 (77)	1.0	
t allele	146 (21)	116 (25)	0.9 (0.7–1.4)	0.85	38 (26)	63 (27)	0.8 (0.5–1.6)	0.60	108 (20)	53 (23)	1.0 (0.6–1.6)	0.91
**VDR-ApaI**												
AA	110 (32)	82 (35)	1.0		28 (38)	49 (43)	1.0		82 (29)	33 (28)	1.0	
Aa	185 (53)	115 (50)	1.0 (0.6–1.7)	0.88	33 (45)	54 (47)	0.8 (0.3–1.8)	0.51	152 (55)	61 (52)	1.3 (0.7–2.4)	0.49
aa	54 (16)	35 (15)	1.1 (0.5–2.1)	0.88	12 (16)	12 (10)	0.6 (0.2–2.2)	0.45	42 (15)	23 (20)	1.3 (0.6–3.0)	0.47
A allele	405 (58)	279 (60)	1.0		89 (61)	152 (66)	1.0		316 (57)	127 (54)	1.0	
a allele	293 (42)	185 (40)	1.0 (0.7–1.4)	0.88	57 (39)	78 (34)	0.8 (0.4–1.4)	0.42	236 (43)	107 (46)	1.2 (0.8–1.7)	0.47

Note: For analysis of alleles F and f, B and b, T and t, A and a, each subject was used twice. **F**- wild type FokI, **f**- polymorphic FokI; **B**- wild type BsmI, **b**-polymorphic BsmI; **T**- wild type TaqI, **t**- polymorphic TaqI; **A**- wild type ApaI, **a**- polymorphic ApaI.

* P-value is significant if P<0.05;

† Analysis adjusted for age, BMI and ethnicity;

†† Analysis adjusted for age and BMI.

Haplotype analysis of the polymorphic variants produced 16 different haplotypes (Table 3). The FBTA (*FokI-F, BsmI-B, TaqI-T and ApaI-A*) was the most common haplotype in Controls and Hispanic/Latina Cases (Table 3). The most common haplotype in African-American Cases was the FbTA haplotype (*FokI-F, BsmI-b, TaqI-T and ApaI-A*). Several VDR-haplotypes were significantly associated with breast cancer in the African-American cohort, however, no association was observed between breast cancer and VDR-haplotypes in the Hispanic/Latina cohort. Logistic regression analysis, using wild-type alleles (FBTA) as the reference category, revealed that FbTA was 1.9 times higher (p = 0.02), FbtA was 1.6 times higher (p = 0.03) and fbtA was 1.4 times higher (p = 0.05) in Cases than in Controls in the African-American cohort (Table 3). Logistic regression analysis performed in Cases showed that African-American women with breast cancer were more likely to have the FbTA (OR = 2.4, p = 0.005) and FbtA (OR = 1.7, p = 0.04) haplotypes compared with Hispanic/Latina women with breast cancer. In contrast to Cases, African-American Controls with the fbTa (OR = 0.8, p<0.001), fbTA (OR = 0.8, p = 0.03), fBTA (OR = 0.8, p = 0.04) and fbtA (OR = 0.7, p = 0.02) haplotypes were significantly less frequently observed than among Hispanic/Latina Controls.

**Table 3:** VDR haplotypes, Breast Cancer, and Ethnicity.

*Association of VDR haplotypes and breast cancer in African-American and Hispanic/Latina women*							
		African-American			Hispanic/Latina		
VDR Haplotypes	Nucleo-tides	Frequencies (%)		Odds Ratio	Frequencies (%)		Odds Ratio
		Cases	Controls	OR∧ (95% CI) *P*	Cases	Controls	OR∧ (95% CI) *P*
FBTA	TGTC	17.0	25.4	1	19.5	16.7	1
FbTA	TATC	26.3	20.6	**1.9 (1.1–3.3) 0.02**	12.4	15.6	0.7 (0.4–1.2) 0.20
FbTa	TATA	7.1	13.4	0.9 (0.8–1.1) 0.53	14.6	11.4	1.0 (0.9–1.1) 0.76
fbTa	CATA	12.1	5.8	1.1 (1.0–1.2) 0.002	16.8	16.4	0.9 (0.9–1.0) 0.65
fbTA	CATC	5.8	5.2	1.1 (0.9–1.4) 0.22	8.0	7.4	0.9 (0.8–1.2) 0.82
FbtA	TACC	7.6	4.5	**1.6 (1.1–2.4) 0.03**	3.1	2.9	0.9 (0.6–1.6) 0.86
FBTa	TGTA	1.8	2.1	1.0 (0.9–1.2) 0.70	2.2	2.7	0.9 (0.8–1.1) 0.57
fBTA	CGTC	1.8	2.1	1.0 (0.8–1.2) 0.70	2.2	4.0	0.9 (0.8–1.1) 0.18
fBTa	CGTA	0.9	0.7	1.0 (0.9–1.2) 0.51	0.9	1.6	0.9 (0.8–1.1) 0.38
fbtA	CACC	4.5	2.4	**1.4 (1.1–1.9) 0.05**	5.8	4.8	1.0 (0.8–1.3) 0.94
FBtA	TGCC	3.1	4.8	1.0 (0.8–1.2) 0.96	3.1	2.9	0.9 (0.8–1.2) 0.86
Fbta	TACA	6.3	4.8	1.1 (0.9–1.1) 0.12	3.1	4.8	0.9 (0.8–1.0) 0.23
fBta	CGCA	0.0	1.7	-	0.9	0.3	1.1 (0.9–1.3) 0.40
fBtA	CGCC	0.0	1.7	-	0.4	1.1	0.8 (0.7–1.2) 0.37
FBta	TGCA	0.4	0.0	-	1.3	0.0	-
fbta	CACA	5.4	4.8	1.0 (0.9–1.1) 0.25	5.8	7.4	0.9 (0.9–1.0) 0.29

*Association of VDR haplotypes and ethnicity in Cases and Controls*							
		Cases			Controls		
VDR Haplotypes	Nucleo-tides	Frequencies (%)		Odds Ratio	Frequencies (%)		Odds Ratio
		AA	Latina	OR* (95% CI) *P*	AA	Latina	OR* (95% CI) *P*
FBTA	TGTC	17.0	19.5	1	25.4	16.7	1
FbTA	TATC	26.3	12.4	**2.4 (1.3–4.6) 0.005**	20.6	15.6	0.9 (0.5–1.4) 0.87
FbTa	TATA	7.1	14.6	0.9 (0.8–1.0) 0.13	13.4	11.4	1.0 (0.9–1.1) 0.36
fbTa	CATA	12.1	16.8	1.0 (0.9–1.1) 0.56	5.8	16.4	**0.8 (0.8–0.9) <0.001**
fbTA	CATC	5.8	8.0	1.0 (0.8–1.2) 0.68	5.2	7.4	**0.8 (0.7–0.9) 0.03**
FbtA	TACC	7.6	3.1	**1.7 (1.0–2.7) 0.04**	4.5	2.9	1.0 (0.6–1.6) 0.99
FBTa	TGTA	1.8	2.2	1.0 (0.9–1.1) 0.91	2.1	2.7	0.9 (0.8–1.0) 0.22
fBTA	CGTC	1.8	2.2	1.0 (0.8–1.2) 0.91	2.	4.0	**0.8 (0.7–1.0) 0.04**
fBTa	CGTA	0.9	0.9	1.0 (0.9–1.2) 0.87	0.7	1.6	0.9 (0.8–1.0) 0.13
fbtA	CACC	4.5	5.8	1.0 (0.7–1.3) 0.81	2.4	4.8	**0.7 (0.6–0.9) 0.02**
FBtA	TGCC	3.1	3.1	1.0 (0.8–1.2) 0.80	4.8	2.9	1.0 (0.9–1.2) 0.86
Fbta	TACA	6.3	3.1	1.1 (0.9–1.2) 0.10	4.8	4.8	1.0 (0.9–1.0) 0.30
fBta	CGCA	0.0	0.9	-	1.7	0.3	1.1 (0.9–1.4) 0.19
fBtA	CGCC	0.0	0.4	-	1.7	1.1	1.0 (0.9–1.2) 0.93
FBta	TGCA	0.4	1.3	0.9 (0.8–1.1) 0.42	-	-	-
fbta	CACA	5.4	5.8	1.0 (0.9–1.1) 0.88	4.8	7.4	**0.9 (0.9–0.99) 0.02**

∧ Cases vs. Controls, Significance is P<0.05;

* African-American vs. Hispanic/Latina ethnicity, Significance is P<0.05.

Table 4 demonstrates the results from linkage disequilibrium (LD) analysis performed on the four VDR variants. The strongest LD is observed between *VDR-TaqI* and *VDR-ApaI* among Hispanic/Latina subjects (D′ = 0.66). Weaker LDs were observed between *VDR-FokI* and the other 3 variants (*VDR-BsmI*, *VDR-ApaI* and, *VDR-TaqI*) in both African-American and Hispanic/Latinas.

**Table 4:** Linkage disequilibrium (LD) between VDR polymorphisms in African-American and Hispanic/Latina women.

	Locus 1	Locus 2	D′ (CI)	LOD	r^2^
African-American	VDRF	VDRB	0.09 (0.00–0.04)	0.06	0.001
	VDRF	VDRA	0.14 (0.02–0.29)	0.56	0.01
	VDRF	VDRT	0.17 (0.00–0.44)	0.21	0.004
	VDRB	VDRA	0.09 (0.00–0.37)	0.07	0.002
	VDRB	VDRT	0.16 (0.03–0.28)	1.01	0.02
	VDRA	VDRT	0.32 (0.07–0.53)	0.94	0.02
Hispanic/Latina	VDRF	VDRB	0.12 (0.00–0.30)	0.27	0.003
	VDRF	VDRA	0.08 (0.00–0.18)	0.58	0.006
	VDRF	VDRT	0.14 (0.01–0.30)	0.30	0.003
	VDRB	VDRA	0.25 (0.08–0.40)	1.48	0.02
	VDRB	VDRT	0.38 (0.27–0.48)	7.80	0.10
	VDRA	VDRT	**0.66 (0.49–0.77)**	8.44	0.09

Note: All samples were in Hardy-Weinberg Equilibrium (HWE) among the groups. LD was calculated between markers among African-Americans or Hispanics/Latinas. D′ is the prime between the loci; LOD is the log of likelihood odds ratio, a measure of confidence in the D'value; r^2^ is the correlation coefficient between the two loci.

The associations between the VDR genotypes and breast tumor histopathology, tumor stage, and metastatic disease progression were assessed in Table 5. The VDR-FokI *FF* genotype was significantly more common in African-American patients than in Hispanic/Latina patients (46.1% vs. 35.9%, respectively, p = 0.02), while the VDR-FokI *ff* genotype was more common in Hispanic/Latina patients as compared to African-American patients (17.1% vs. 6.1%, respectively). African-American patients were more likely to have VDR-ApaI *AA* genotype and Hispanic/Latina patients were likely to have VDR-ApaI *Aa* or *aa* genotypes (p = 0.008). There was also a significant association identified between VDR-ApaI polymorphisms and tumor differentiation (p = 0.04). Poorly differentiated tumors were more likely to express a polymorphic allele of VDR-ApaI (*Aa* or *aa*). There were no other significant associations found between any of the polymorphic VDR variants and tumor stage, tumor differentiation, and ER/PR/HER2 receptor status.

**Table 5:** Association of VDR genotypes with Tumor Pathology and Ethnicity.

	VDR-FokI			VDR-BsmI			VDR-TaqI			VDR-ApaI		
	FF	Ff	ff	BB	Bb	bb	TT	Tt	tt	AA	Aa	aa
**Ethnicity**												
AA	46%	48%	6%	8%	35%	57%	57%	30%	12%	43%	47%	10%
Latina	36%	47%	17%	9%	43%	49%	64%	27%	9%	28%	52%	20%
	**p = 0.02**			p = n.s.			p = n.s.			**p = 0.008**		
**ER/PR Status**												
ER/PR+ve	42%	47%	11%	8%	41%	51%	59%	29%	12%	36%	49%	15%
ER/PR -ve	42%	46%	12%	6%	39%	55%	62%	25%	13%	35%	51%	14%
	p = n.s.			p = n.s.			p = n.s.			p = n.s.		
**HER2 Status**												
HER2 +ve	40%	55%	5%	11%	40%	50%	63%	21%	16%	42%	45%	13%
HER2 -ve	42%	45%	13%	7%	40%	54%	60%	28%	11%	36%	52%	12%
	p = n.s.			p = n.s.			p = n.s.			p = n.s.		
**Distant Metastasis**												
Yes	44%	56%	0%	11%	33%	56%	56%	22%	22%	33%	33%	33%
No	41%	47%	12%	7%	40%	53%	61%	28%	11%	37%	48%	15%
	p = n.s.			p = n.s.			p = n.s.			p = n.s.		
**Differentiation**												
Well	44%	33%	22%	0%	44%	56%	56%	44%	0%	67%	33%	0%
Moderate	34%	51%	15%	7%	53%	41%	59%	31%	10%	33%	61%	7%
Poor	44%	47%	9%	8%	38%	55%	61%	24%	16%	34%	46%	20%
	p = n.s.			p = n.s.			p = n.s.			**p = 0.04**		
**Stage**												
0	53%	33%	13%	13%	27%	60%	60%	40%	0%	40%	27%	33%
Ι	39%	48%	13%	10%	32%	58%	55%	36%	10%	32%	48%	19%
ΙΙ	39%	50%	12%	5%	42%	53%	63%	24%	13%	41%	47%	12%
ΙΙΙ	46%	47%	8%	6%	43%	51%	65%	24%	12%	31%	55%	14%
ΙV	36%	46%	18%	9%	36%	55%	46%	27%	27%	36%	36%	27%
	p = n.s.			p = n.s.			p = n.s.			p = n.s.		

Note: N.s. is not-significant with a P-value>0.05. Significance is P<0.05.

The 5-year disease-free-survival (DFS) from breast cancer in association with VDR polymorphisms is shown in Figure 1. The 5-year DFS in patients carrying VDR-FokI *FF* genotype is reduced significantly compared to VDR-FokI *Ff* and *ff* genotypes (p = 0.05). The VDR-BsmI, VDR-ApaI and VDR-TaqI polymorphisms did not influence DFS significantly. Results of multivariate analyses, adjusted for the tumor characteristics, ethnicity, and the four VDR polymorphic variants, confirm the independent predictor value of VDR-FokI in DFS as shown in Table 6. The relative risk of tumor recurrence or metastases was decreased by 43% in patients who had the polymorphic VDR-FokI alleles, *Ff* or *ff*, compared to subjects who had VDR-FokI *FF* genotype (Table 6).

**Figure 1:** Five-year disease free survival (DFS) of breast cancer patients in relation to VDR gene polymorphisms. Kaplan-Meier survival curves were used to compare the 5-year DFS between the VDR gene polymorphisms in (a) VDR-FokI, (b) VDR-BsmI, (c) VDR-ApaI, and (d) VDR-TaqI. The differences between the curves were estimated by log-rank test, where P<0.05 was considered statistically significant.

**Table 6:** Relative Risk of worse Disease-Free-Survival in relation to VDR gene polymorphisms (Multivariate Analysis).

Polymorphism	RR*	(95% CI)	*P*-value
**FokI**			
FF	**1**	**(0.3–0.9)**	**0.05**
Ff+ff	**0.57**		
**BsmI**			
BB	1	(0.3–1.9)	0.45
Bb+bb	0.67		
**ApaI**			
AA	1	(0.5–1.7)	0.80
Aa+aa	0.92		
**TaqI**			
TT	1	(0.7–2.4)	0.48
Tt+tt	1.3		

* RR: Relative Risk adjusted for tumor characteristics and ethnicity.

## Discussion

The results from our study reveal an increased association between one of the VDR polymorphic variants, VDR-FokI, and breast cancer in the African-American cohort. The odds ratio (OR) for breast cancer in association with the VDR-FokI *f* allele was 1.9 (95% CI = 0.9–3.7; p = 0.07). This is consistent with other studies [25] which have identified a positive association between the VDR-FokI *ff* genotype and/or *f* allele and breast cancer (Table 7). Our study further identifies that this trend is present among African-American women, but not Hispanic/Latina women. The other most commonly studied VDR polymorphism, VDR-BsmI, was not associated with breast cancer in our study, similar to most of the other studies conducted on this polymorphism (Table 7). While Ingles *et al* [14] identified a significant association of the *B* allele with breast cancer among Hispanics, recent large studies and meta-analyses on various ethnic groups, including Hispanics, have suggested otherwise. For example, the large analyses conducted by Rollison *et al* [19] and Tang *et al* [10] have confirmed that there is no significant association between VDR-BsmI and breast cancer. Furthermore, data from our current study shows no associations between the two other VDR variants (TaqI and ApaI) and breast cancer, consistent with most studies to date on Caucasian populations (Table 7). The VDR-TaqI (*tt* genotype) and VDR-ApaI (*a* allele) were significantly associated with breast cancer in only two hospital-based studies [15], [16]. However, these polymorphisms were found to be non-significant in recent large population meta-analyses [10]. Linkage-disequilibrium analysis of the polymorphisms in our study is also consistent with findings from previous studies, confirming linkage between VDR-TaqI and VDR-ApaI in Hispanic/Latina women, and absence of LD between the VDR-FokI and other SNPs [6].

**Table 7:** Summary of Studies on Breast Cancer and VDR polymorphisms.

*Reference*	*Study design*	*Ethnicity*	*No. of Cases*	*No. of Controls*	*Association between VDR polymorphism and breast cancer*			
					*FokI*	*BsmI*	*TaqI*	*ApaI*
Curran, 1999 [16]	Hospital	Caucasian	135	110	*n.s.*		*n.s.*	*a allele*
Dunning, 1999 [27]	Hospital/Population	Caucasian	951	627			*n.s.*	
Ingles, 2000 [14]	Population	Latinas	143	300	*n.s.*	*B allele*		
Bretherton-Watt, 2001 [28]	Hospital	Caucasian	181	241	*n.s.*	*bb type*		
Guy, 2004 [17]	Hospital	Caucasian	398	427	*n.s.*	*bb type*		
Hefler, 2004 [29]	Hospital/Population	Caucasian	390	1,699		*n.s*		
Chen, 2005 [30]	Population	Caucasian	1,234	1,676	*ff type*	*n.s.*		
Vande Vord, 2006 [31]	Hospital	Mixed	220	192		*n.s.*		
		Caucasian (50.3%)						
		AA(49.7%)						
John, 2007 [32]	Population	Mixed	1,786	2,127	*n.s.*	*n.s.*	*n.s.*	
		Caucasian	596	646				
		AA	543	598				
		Hispanic	647	883				
McCullough, 2007 [15]	Population	Caucasian	500	500	*n.s.*	*n.s.*	*n.s.*	*n.s.*
Trabert, 2007 [21]	Population	Caucasian	1,143	987		*bb type* *		
		AA	488	448		*n.s.*		
Abbas, 2008 [26]	Population	Caucasian	1,403	2,609	*n.s.*		*n.s.*	
Gapska, 2008 [33]	Population	Caucasian	800∧	550	*f allele*	*n.s.*	*n.s.*	
Sinotte, 2008 [34]	Hospital/Population	Caucasian	859	1,381	*ff type*	*n.s.*		
Barroso, 2008 [35]	Hospital	Caucasian	549	556	*ff type* #		*tt type* a	
McKay, 2009 [25]	Population	Caucasian	378	421	*n.s.*	*n.s.*		
		AA	325	419	*n.s.*	*n.s.*		
		Hispanic	318	378	*n.s.*	*n.s.*		
		Asian	401	405	*ff type*	*Bb type^a^*		
		Hawaiian	104	278	*n.s.*	*n.s.*		
Tang, 2009 [10]	Meta-Analysis	All ethnicities	>5,000	>7,000	*ff type*	*n.s.*	*n.s.*	*n.s.*
Raimondi, 2009 [9]	Review	All ethnicities	14,863	21,318	*ff type*	*n.s.*		
Rollinson, 2012 [19]	Population	Non-Hispanic White	1,527	1,599	*n.s*	*n.s.*		
		Hispanic	791	922				
Vadgama, 2012	Hospital	AA	115	73	*f vs. F, OR = 1.9, p = 0.07*	*n.s.*	*n.s.*	*n.s.*
		Latina	117	267	*n.s.*	*n.s.*	*n.s.*	*n.s.*

AA: African-American.

* for postmenopausal women.

∧ for early-onset breast cancer (age<50).

# OR adjusted for age at diagnosis, number of live births, age at menarche and menopause.

a associated with low risk of breast cancer.

Additional studies on VDR SNPs [26]–[35] are presented in Table 7. Abbas *et al* [26], suggested that VDR polymorphisms may affect postmenopausal breast cancer risk, and be associated with receptor status. Our study shows no receptor-specific association (ER/PR/HER +/−) with any of the VDR polymorphic variants; however, the VDR-ApaI *aa* genotype is significantly associated with poorly differentiated tumors (p = 0.04). Since the VDR-ApaI *a* allele is most common in Hispanic/Latinas, and the Latinas in the present study were slightly younger than the African-American subjects, these findings may potentially implicate VDR-ApaI in the progression of cancer among younger breast cancer patients. Further investigation among larger numbers of younger women with breast cancer is necessary in order to discern a definite association.

Lastly, recent reviews have concluded that the scientific evidence between vitamin D status and breast cancer risk and outcome are fairly strong, and improving vitamin D levels could improve health status [36]. Unfortunately, studies to date which have utilized vitamin D supplementation to overcome vitamin D insufficiency have not yielded conclusive improvements in cancer health risks and outcomes [37], [38]. Hence examination of the Vitamin D receptor (VDR), and genetic changes such as polymorphisms potentially impacting VDR protein function may be central in identifying confounding factors that play a role in Vitamin D activity and ultimately patient outcome. Our study identifies that the 5-year disease-free-survival from breast cancer is significantly reduced among breast cancer patients with the VDR-FokI *FF* genotype (Log rank = 6.06 and p = 0.05). Cox regression with multivariate analysis demonstrates the independently predictive value of VDR-FokI on DFS. Hence, findings from our study suggest that while the VDR-FokI *f* allele may play a role in early association with breast cancer development, the *F* allele may play a role on tumor progression and patient outcome. The findings on these VDR variants, together with significant differences in haplotypes between Cases and Controls suggest the potential need to screen for VDR polymorphisms in the context of breast cancer, particularly before considering Vitamin D supplementation.
